RETRACTED

# A pedagogical approach for the development and optimization of a novel mix of biowastes-derived hydroxyapatite using the Box-Behnken experimental design

**DOI:** 10.1016/j.heliyon.2023.e23092

**Published:** 2023-12-03

**Authors:** Obinna Anayo Osuchukwu, Abdu Salihi, Ibrahim Abdullahi, Bello Abdulkareem, Kazeem Adeniyi Salami, Precious Osayamen Etinosa, Solomon C. Nwigbo, Sikiru Adepoju Mohammed, David Olubiyi Obada

**Affiliations:** a Department of Mechanical Engineering, Bayero University, Kano, 700241, Kano State, Nigeria; b Department of Mechanical Engineering, Ahmadu Bello University, Zaria, 810222, Kaduna State, Nigeria; c Department of Mechanical Engineering, Worcester Polytechnic Institute, 100 Institute Road, Worcester, MA, 01609, USA; d Department of Mechanical Engineering, Nnamdi Azikiwe University, Awka, 420007, Anambra State, Nigeria; e Mechanical Engineering Department, Nigerian Defence Academy, PMB 2109, Kaduna, Nigeria; f Multifunctional Materials Laboratory, Shell Chair Office in Mechanical Engineering, Ahmadu Bello University, Zaria, 810222, Kaduna State, Nigeria; g Africa Centre of Excellence on New Pedagogies in Engineering Education, Ahmadu Bello University, Zaria, 810222, Kaduna State, Nigeria

**Keywords:** Calcination, Mechanical property, Porosity, Sol-gel, Sintering temperature, Engineering education

## Abstract

The current study details the creation of synthetic hydroxyapatite (HAp) using a combination of catfish and bovine bones (C&B). This is done to design the optimum processing parameters and consolidate instructional strategies to develop HAp scaffolds for biomedical engineering. The HAp produced from the novel mix of the biogenic materials (C&B) was through calcination and supported with the sol-gel technique, sintering, and low-cold compaction pressure. The ideal preparation conditions were identified with the aid of the Box-Behnken statistical design in response surface methodology. To understand the physicochemical and mechanical properties of the formulation, analytical studies on the synthesized HAp were carried out. To establish a substantial relation between the physicomechanical properties of the produced HAp scaffolds, three parameters— sintering temperature, compaction loads, and holding times were used. In the evaluation, the sintering temperature was found to have the greatest impact on the material's physicomechanical properties, with compressive strength (13 MPa), porosity (49.45 %), and elastic modulus (2.216 GPa) being the most enhanced properties in that order. The physicomechanical characteristics of the HAp scaffolds were at their optimal at 900 °C, 1 h 18 min of holding time, and 311.73 Pa of compaction pressure. X-ray diffraction (XRD) and Fourier transform infrared (FTIR) results showed that powders with a dominant HAp phase were produced at all runs, including the optimum run. Therefore, using a computationally effective methodology that is helpful for novelties in biomedical engineering education, this study demonstrates the optimal process for the synthesis of a novel matrix bone-derived HAp, showing the most significant relations liable for manufacturing medically suitable HAp scaffolds from the mixture of bovine and catfish bones.

RETRACTED

## Abbreviations

ANOVA: Analysis of Variance
BI: Brittleness Index
CC: Coefficient of Correlation
BBD: Box-Behnken Design
BBED: Box-Behnken Experimental Design
DTA: Differential Thermal Analysis
EDS: Energy Dispersive Spectroscopy
FTIR: Fourier Transform Infrared
HAp: Hydroxyapatite
PBS: Phosphate Buffer Saline
RF: Response Factors
RSM: Response Surface Methodology
SD: Standard Deviation
SEM: Scanning Electron Microscopy
TGA: Thermogravimetric Analysis
UTM: Universal Testing Machine
XRD: X-Ray Diffraction

## 1 Introduction

Hydroxyapatite (HAp), which has high mechanical strength, has several potential applications in orthopedics and dentistry, drug delivery, filling bone defects, creating bone cement, and other biomedical engineering applications [[1], [2], [3]]. HAp exhibits high biocompatibility and chemical similarity to natural bone [4,5,]. To meet the demands of the biological application, however, the handling of pure HAp must appropriately address its low mechanical integrity, which is a drawback [6]. The ideal implant is crucial for bioactivity and relative mechanical reliability [[7], [8], [9]]. Research has concentrated on producing HAp bio-ceramics using a range of processing methods to achieve this. It is important to note that producing HAp materials from natural sources offer the opportunity to reduce waste pollution and it is affordable, friendly, and environmentally sustainable because of the abundance of natural biowastes, with low-cost techniques to prepare industrially useful ceramic materials [7,[10], [11], [12], [13], [14], [15], [16], [17], [18], [19]]. It has been established that the conventional sintering technique is an easy and inexpensive way to produce HAp powder from biogenic sources and to produce ceramic compacts at a competitive price [20,21]. Some of these processes have been used in the production of HAp. Although the physical and mechanical properties of the materials and structures in these designs are well established, there is still little knowledge of the structure-property relationships and the interaction and mechanistic complexities necessary for robust material design and process optimization.

RETRACTED

In the context of research, study, and training, the resolution of a collection of scientific problems can be achieved using various mathematical approaches [20]. The complexity of research findings can be made more difficult by several elements that analytical devices can create in large quantities. This facilitates the establishment of a methodology for the selection, arrangement, and implementation of statistical analyses about experimental components [21,22]. In this context, the utilization of response surface methodology (RSM), a specific experimental design approach, might offer benefits in optimization endeavours where multiple variables have the potential to influence the product. The HAp used in this investigation was synthesized using a combination of calcination, sol-gel methodology, conventional sintering, and low compaction pressure, as described in Ref. [23]. Hence, the utilization of RSM holds significance within this context as it enables the assessment of how the collective impacts of various aspects can be leveraged to enhance the efficiency of HAp production and processing, thereby reducing operational downtime [24]. The Box-Behnken design (BBD) is a second-order approach inside the RSM framework. It utilizes incomplete factorial designs with three layers and has rotatable or nearly rotating properties [25]. The Box-Behnken Experimental Design (BBED) in RSM has been documented as superior to other 3-level designs when analyzing measurable variables due to its ability to collect data points from the 3-level factorial plan [[25], [26], [27]].

Sen et al. [28] produced HAp from eggshells using the biosorption technique to the applicability of glyphosate (GLY) elimination from the aqueous phase. BBED was employed to study the influence of the biosorption process. They concluded that the adsorbent usefulness can be favorable to the adsorption of GLY in sustainable techniques. Go et al. [29] used RSM to design and optimize the degradation efficiency parameter after the HAp photocatalyst degraded levofloxacin. The reaction was fixed into a two-factor interface equation, and the ANOVA calculation was reported as R^2^ = 97.08 %, and adjusted R^2^ = 94.89. Kehoe & Stokes [30] created HAp using a chemical precipitation process from biowaste(s). To determine the ideal set of process parameters and their impact on various HAp properties, a BBD 3-level experimental technique was chosen. According to this research, the ideal characteristics for HAp powder used in orthopedics and applied with the thermal spray technique can be achieved through specific chemical precipitation process parameters. Thomas et al. [31] prepared nano-HAp and optimized the process using BBED. Remarkable results were obtained based on in vitro, in vivo, and analytical studies. Using the BBED process, Dizaj et al. [32] prepared and optimized ciprofloxacin hydrochloride loaded-CaCO_3_ nanoparticles using BBED. They proposed that the BBED is an effective technique for improving drug-incorporated calcium carbonate nanoparticles. Kavitha et al. [33] produced a strontium-substituted HAp using the solution combustion technique. To investigate the key development variables, Box-Behnken was utilized. Their findings demonstrated that the 3 characteristics expressively impacted the response variables. The temperature of 500 °C for 30 min enhanced the size of the crystallites containing the percent (%) Sr substitution, resulting in the maximum yield.

RETRACTED

The BBED frequently supports predicting the cause-and-influence connection between response factors and dependent variables, thus saving a great deal of time. Numerous studies have sought to improve the various treating conditions to produce HAp powders that are helpful for both industrial and medicinal purposes [[34], [35], [36], [37], [38], [39]]. The Taguchi approach was used in an earlier study [40] to improve three novel mixed samples made from animal wastes. The sample with 50 g of bovine (B50) and 50 g of catfish (C50) bones was the ideal sample (B50/C50) with the optimal processing characteristics according to the results. In comparison to other experimental designs, it is reckoned that the BBED is a useful and economical tool for this study to compare the reported results [40] and suggest the optimum parameters for learning to produce natural HAp with improved mechanical properties. From the standpoint of HAp synthesis, chemical sedimentation, hydrolysis processes, sol-gel, hydrothermal techniques, etc. are examples of wet reaction techniques. Wet techniques are therefore interesting ways to produce nanoparticles because they offer control over the size and shape of the particles [41]. Acceptable purity [40], controlled size and shape [42], ability to produce uniform materials [43], as well as easy-to-use and affordable equipment [44] are other potential advantages of the sol-gel technique over others. Bakhtiari et al. [45] used a sol-gel approach to produce 80S bioactive glasses with different Ca/P ratios. The HAp nanoparticles' production is controlled by several factors. To find the ideal synthesis conditions, numerous tests and a lot of time are needed [46]. The manufacture of HAp nanoparticles with desirable characteristics depends heavily on variables including sintering temperature[47], compaction load, and holding time or duration. For the first time, we report the adoption of the BBD optimization approach in this work to determine the ideal preparation conditions for HAp made from a combination of bovine and catfish bones.

RETRACTED

It is important to emphasize the value of instructional research in computational bioengineering training from the standpoint of knowledge transfer. For hands-on learning, it is essential to adopt instructional approaches that can be applied anywhere, even in developing laboratories. In this article, we propose an approach to contribute to the database on the synthesis and characterization of a specific mixture of biowaste-derived HAp scaffolds. This method builds on existing techniques while creating new perspectives [39].

Therefore, in the current study, considering the B50/C50 sample [40], we show how the sintering temperature, compaction load, and holding time interact with one another to produce a mixture of HAp produced from catfish and bovine bones utilizing the BBED. We predict that sintering temperature substantially impacts the mechanical and physical properties of HAp powders since it increases the phase stability of HAp. In contrast, the compaction strength, porosity, and density of HAp are affected by the compaction pressure, whereas the coalescence of the material which impacts its mechanical properties like brittleness index, hardness, and porosity, is significantly influenced by the holding time. The optimization of these parameters serves as a reference for choosing the three parameters in producing a new blend of HAp from bovine and catfish bones derived biowastes for biomedical uses and instructional purposes. From the results obtained, the complexity of producing an innovative blend of HAp from other sources can be reduced. The ideal process parameter settings for the development of medically useful HAp are identified in this research.

## 2 Materials and methods

Bovine bones were obtained from an abattoir located in the Zaria metropolitan region, Nigeria, whereas catfish bones were collected from local restaurants in the same vicinity. The bones underwent deproteinization by the utilization of a specifically designed oven. The synthesis of HAp powders has been documented in our recent articles [[48], [49], [50], [51], [52], [53]]. Following the calcination process, the powders derived from the two sources were carefully measured and subsequently combined using a spatula in varying ratios to obtain a total mass of 100 g, specifically consisting of 50 g of bovine bones and 50 g of catfish bones. The powder mixture consisting of bovine and catfish bones was subjected to individual calcination processes at different temperatures (700, 800, and 900 °C) using a muffle furnace. The calcination duration for each temperature was either 1 or 2 h. Subsequently, the bones devoid of proteins from both sources were subjected to crushing and subsequent sieving using a 100 μm sieve. The specimens were subjected to pelletization using a low compaction pressure of 300, 400, and 500 Pa to facilitate mechanical measurements. The microhardness of the samples was evaluated using Vickers' microhardness tester. The evaluation of the compressive strength of the fabricated scaffolds was conducted using a universal testing machine (UTM) [54]. The fracture toughness, denoted as KIC, was determined by employing the parameters of the hardness test, as indicated in Ref. [55]. The evaluation of the brittleness index was conducted per the methodology outlined in Ref. [55]. The elastic modulus was determined through indentation using a TI 950 Hysitron Tribo-Indenter (Bruker Instruments, Minneapolis, MN) equipped with a Berkovich tip. The indentation investigations were carried out under controlled conditions with a consistent room temperature of 25 °C. The determination of the elastic modulus followed the methodology outlined in Ref. [56]. The formula referenced in Ref. [57] was utilized to compute the porosity and density of the produced HAp, hence determining its physical parameters. To assess the thermal stability of the powders, a simultaneous thermogravimetric analysis/differential scanning calorimetry (TGA/DSC) was conducted utilizing a SDT Q600 instrument. The thermal analysis was conducted at a constant heating rate of 20 °C per minute up to a temperature of 1200 °C.

RETRACTED

### 2.1 Optimization

The design simulations and experiments were conducted using the Software Design Expert® 13.0. The research contained three separate independent variables, specifically heating temperatures, compaction load, and holding duration. The minimum and maximum values for each variable are displayed in Table 1. The identification of the optimal combination of processing variables to produce clinically viable HAp was accomplished by employing a BBED with three levels and three components. The independent variables adjusted in this experimental design included sintering temperature (A), compaction load (B), and holding time (C). The results linked to the interaction of the independent variables included hardness, fracture toughness, brittleness index, compressive strength, elastic modulus, porosity, and density. Based on the data shown in Table 2, a cumulative count of 14 experimental trials was proposed. The conditions were carefully utilized to examine the effects of independent factors on the structural and mechanical characteristics of the HAp based materials. Numerous studies have been undertaken to examine the elements that contribute to the reduced mechanical properties of HAp [1,2,[7], [8], [9],^19^,^58^]. Numerous investigations have repeatedly demonstrated that the predominant factor contributing to this problem is the usage of elevated sintering temperatures and extended holding durations in the manufacturing process. The conditions frequently give rise to insufficient grain enhancements and non-uniform microstructures, hence leading to reduced mechanical properties of HAp. Therefore, the determination of design temperatures was influenced by prior research that suggested the requirement of temperatures below 900 °C for the synthesis of HAp, while also ensuring adequate porosity, to promote the rapid proliferation of cells [18,20]. The determination of the optimal preparation parameters was carried out by employing a third-order polynomial function generated from the experimental design. The traditional polynomial equation (Eqn. (1)) was employed to establish the relationship between input and target values, as proven in previous studies [14,59,60].

(1) $$Y_{i}=\alpha_{0\;}+\alpha_{1\;}A+\alpha_{2\;}B+\alpha_{3\;}C+\alpha_{4\;}AB+\alpha_{5\;}BC+\alpha_{6\;}AC+\alpha_{7\;}A^{2}+\alpha_{8\;}B^{2}+\alpha_{9\;}C^{2}+\alpha_{10\;}ABC+\alpha_{11\;}A^{2}B+\alpha_{12\;}A^{2}C+\alpha_{13\;}AB^{2}+\alpha_{14\;}AC^{2}+\alpha_{15\;}B^{2}C+\alpha_{16\;}BC^{2}+\alpha_{17\;}A^{3}+\alpha_{18\;}B^{3}+\alpha_{19\;}C^{3}+\alpha_{20\;}A^{2}B^{2}+\alpha_{21\;}A^{2}B+\varepsilon \;$$

In equation (3), the symbol Yi represents the anticipated response, while A, B, and C denote the independent factors under investigation. The constants and coefficients of the equation are represented by α_1_ – α_21_, and the symbol ℇ represents the slip that is obtained. The statistical parameters were determined by employing an analysis of variance (ANOVA). The statistical significance level of all mechanical and physical level outcomes was assessed by examining a p-value of <0.05. The F-test (Ft) and coefficient R^2^ were employed to evaluate the degree of appropriateness of the trial outcomes inside the polynomial model equation, hence indicating the goodness or lack of fit. The significance of each term in the polynomial equation [[31], [32], [33], [34],^39^] was determined using the Ft within a 95 % confidence interval.

RETRACTED

**Table 1:** Optimization approach.

Factors	Code	Units	Type	Lowest	Highest
A	Sintering Temperature	^o^C	Numeric	700	900
B	Compaction Load	Pa	Numeric	300	500
C	Holding Time	Hours	Numeric	1	2

**Table 2:** Box Behnken Experimental conditions for optimization study.

Exp. Run	A: Heating Temp (^o^C)	B: Compaction Load (Pa)	C: Holding Duration (Hours)	Response(s)
1	800	500	1	
2	700	500	1.5	
3	800	300	2	
4	700	300	1.5	
5	900	400	2	
6	800	500	2	
7	700	400	2	
8	800	300	1	
9	900	300	1.5	
10	700	400	1	
11	900	400	1	
12	900	500	1.5	
13	800	400	1.5	
14	800	400	1.5	

## 3 Characterization of the produced HAp

3

The produced HAp powders used in the experimental trials (as shown in Table 3) were subjected to characterization using Fourier-transform infrared spectroscopy (FT-IR) and X-ray diffraction (XRD) techniques, as described in Ref. [49]. The morphology of the HAp obtained, consisting of a mixture of B50 and C50, as well as the individual powders of B and C, was examined using scanning electron microscopy (SEM) at an accelerating voltage of 20 kV. The powders from run 6, which represented the optimum sample run, were also included in the analysis. The investigation of the biodegradability of the run 6 sample was conducted by immersing the pellets in a solution of phosphate buffer saline (PBS).

**Table 3:** Actual Box-Behnken experimental design.

Order	Run	HT (^o^C)	CP (Pa)	HT (Hrs)	H (GPa)	CS (MPa)	FT (MPa.m^1/2^)	BI	PO (%)	DE (Kg/m^3^)	EM (GPa)
10	1	800	500	1	0.37	11	0.05	5.5	54.96	1.89	0.06
3	2	700	500	2	0.36	10	0.05	4.8	51.38	1.86	0.84
11	3	800	300	1.5	0.38	17	0.04	6.4	53.69	1.59	0.72
1	4	700	300	1.5	0.35	18	0.06	7.2	45	1.88	4.2
8	5	900	400	2	0.38	11	0.07	5.8	44.06	1.89	4.37
12	6	800	500	1.5	0.37	12	0.06	5.7	46	1.86	0.84
7	7	700	400	2	0.23	11	0.05	4.8	48.7	1.89	4.21
9	8	800	300	1.5	0.2	10	0.05	4.4	49.72	1.58	0.06
2	9	900	300	2	0.26	8	0.04	7.1	48.95	1.86	0.73
5	10	700	400	2	0.38	15	0.06	6.1	53.96	1.82	4.37
6	11	900	400	1	0.41	17	0.07	6	52.6	1.81	4.21
4	12	900	500	1.5	0.37	17	0.06	5.8	50.44	1.87	0.84
13	13	800	400	1	0.34	10	0.07	5.1	45.88	1.88	4.12
14	14	800	400	1.5	0.32	11	0.06	5.3	47.33	1.87	4.34

HT = Heating Temperature; CP = Compaction Pressure; HT = Heating Duration; H = Hardness; CS = Compressive Strength; FT = Fracture Toughness; BI = Brittleness Index; PO = Porosity; DE = Density and EM = Elastic modulus.

## 4 Results and discussion

### 4.1 Synthesis of HAp

In this work, bovine and catfish bones were used to produce HAp via a sol-gel synthesis process [59]. The technique enabled the development of a novel mix of powders with a dominant HAp phase.

### 4.2 Thermal analysis results

The DTA curves of the synthetic HAp powders have four areas in both bovine and catfish bone samples (Fig. 1 (A) and (B)). Based on the corresponding trend generated from the TGA data, these four zones can be given. The weight loss for DTA in Region I correlated with the loss of water contained in the HAp samples. At 458 °C, Region II exhibits an endothermic peak. Region III underwent little alterations, whereas Region IV experienced a slight weight decrease and this is in line with research elsewhere [61]. At 254.10 °C, a significant weight loss was noticed from the evaporation of absorbed water, and at 884.50 °C, there was just a little loss of weight. At 1200 °C, no significant loss was detected. Within the temperature range, stable curvature was noticed, demonstrating the thermal stability of the produced HAp powders [62,63].

RETRACTED

**Fig. 1:** Thermal analysis of the bones: (A) Catfish & (B) bovine.

### 4.3 Results from the optimization

The BBED gave 14 experimental trials, as described in the method section (i.e., section 2.1), and the results are displayed in Table 3. The findings demonstrate that:

• The design parameters promote the HAp's good mechanical and physical properties. As fracture toughness yielded values greater than 0.04 MPa m^1/2^ (Runs 1–8, and 10–14), and compressive strength ranged from 8 to 18 MPa.
• The densification of HAp increased at higher sintering temperatures with high compaction load because of quick crystal border movement and blend of increasing and more refined grain borders, which increased compressive strength [64] with less porosity.
• Increased mechanical characteristics of pelletized ceramic pellets have been shown to benefit from higher sintering temperatures [19,65,66].
• According to the ANOVA report, the sintering temperature (A) demonstrates the highest level of significance across all response factors. Additionally, the compaction load (B) and holding duration (C) show significance for the response variables of hardness value, compressive strength, fracture toughness, and elastic modulus. This finding is consistent with the results of research conducted by Ref. [46].

Table 4 describes observations as follows:

• The compressive strength, fracture toughness, porosity, and density are all affected by the 2nd-order variables for sintering temperature (A^2^), whereas holding time (B^2^) had an impact on hardness and compressive strength.
• Table 4 presents a comprehensive display of significant statistical metrics that can be employed to ascertain the elevated level of predictability shown by the models. The initial observation pertains to the narrow standard deviation (SD) of the response data, which serves as an indicator of the degree of similarity between the observed values and the fitted values. Lower standard deviation (SD) values indicate that the model has a higher level of accuracy in predicting the responses. The statistical correlation coefficients (R^2^), which quantify the proportion of variance in responses explained by the model, demonstrated values that approached unity. The values in question exhibit a high degree of stability within the model, as evidenced by their consistent presence in Table 4. Furthermore, these values surpass the corresponding value reported in a previous study [39]. The model's appropriateness increased as the value of R^2^ approached 1.
• All of the response factors' non-significant Lack of Fit p-values concerning the slips indicate that the models are accurate and adequate for the experiments.
• Except for the hardness & fracture toughness, which divergence can be attributed to real design values, all the models in Table 3 have appropriate precision ratios greater than 2. This explains the model discrimination's suitability and the design trials' adequate navigation [39,60].

RETRACTED

**Table 4:** Statistical pointers of the model.

Serial	RF	SD	CC (R^2^)	MS (p-value)	Non-significant lack of Fit (p-value)	Adequate precision ratio
1	Hardness	0.0387	0.7083	0.0050	0.1341	0.3515
2	Compressive strength	0.7906	0.9827	0.0041	0.0274	23.0227
3	Fracture toughness	0.0071	0.5833	0.0274	0.0734	0.0924
4	Brittle index	0.8847	0.7700	0.2861	0.3497	9.5465
5	Porosity	3.5320	0.5767	0.3277	0.4630	64.6622
6	Density	0.1045	0.6445	0.8462	0.9464	2.2743
7	Elastic Modulus	1.3733	0.7257	0.0249	0.0438	9.4748

**RF-** Response Factors; **SD** – Standard deviation; **CC**- Coefficient of Correlation, **MS** – Model Significance.

### 4.4 Situation study Diagnostics/analysis

The outcomes of the diagnostic situation studies for the corresponding response factors are presented in Table 5. The results of the experiments are reflected by the actual values in the table, whilst the anticipated values show the outcomes of the design and experimental analysis (BBED Model).

• The degree of model accuracy is indicated by how closely the values obtained from experiments match the predicted values, also known as residuals [29].
• The constant predicted value in the brittleness index is 5.7.
• Positive residual data indicate that the estimated value is more than the observed value, whereas negative residual data suggest that the observed value is greater than the estimated value. When the residual value is equal to zero, the actual value aligns with the anticipated value that was employed as the foundation for the comparison.

**Table 5:** Incident study diagnostic for actual and predicted.

Order	H (GPa) A P	CS (MPa) A P	FT (MPa.m^1/2^) A P	BI A P	PO (%) A P	DE (Kg/m^3^) A P	EM (GPa) A P
10	0.37 0.40	11 11	0.05 0.05	5.5 5.7	54.96 49.48	1.89 1.82	0.06 0.74
3	0.36 0.36	10 10	0.05 0.05	4.8 5.7	51.38 49.48	1.86 1.82	0.84 0.19
11	0.38 0.38	17 17	0.04 0.05	6.4 5.7	53.69 49.48	1.59 1.82	0.72 2.42
1	0.35 0.35	18 18	0.06 0.06	7.2 5.7	45.00 49.48	1.88 1.82	4.20 4.60
8	0.38 0.38	11 11	0.07 0.07	5.8 5.7	44.06 49.45	1.89 1.82	4.37 4.73
12	0.37 0.37	12 12	0.06 0.06	5.7 5.7	46.00 49.48	1.86 1.82	0.84 0.94
7	0.23 0.26	11 11	0.05 0.05	4.8 5.7	48.70 49.48	1.89 1.82	4.21 3.38
9	0.20 0.25	10 10	0.05 0.05	4.4 5.7	49.72 49.48	1.58 1.82	0.06 0.82
2	0.26 0.26	8 8	0.04 0.04	7.1 5.7	48.95 49.48	1.86 1.82	0.73 0.13
5	0.38 0.38	15 15	0.06 0.06	6.1 5.7	53.96 49.48	1.82 1.82	4.37 4.73
6	0.41 0.40	17 17	0.07 0.07	6.0 5.7	52.60 49.48	1.81 1.82	4.21 3.28
4	0.37 0.41	17 17	0.06 0.06	5.8 5.7	50.44 49.48	1.87 1.82	0.84 2.42
13	0.34 0.34	10 10	0.07 0.07	5.1 5.7	45.88 49.48	1.88 1.82	4.12 4.10
14	0.32 0.32	11 11	0.06 0.07	5.3 5.7	47.33 49.48	1.87 1.82	4.34 4.02

**A = Actual value and P = Predicted value.** H = Hardness; CS = Compressive Strength; FT = Fracture Toughness; BI = Brittleness Index; PO = Porosity; DE = Density and EM = Elastic modulus.

RETRACTED

The quadratic polynomial model was employed to fit the data, using various statistical factors. After conducting data modeling, polynomial equations (2.1–2.7) were generated, which demonstrated the presence of interaction and curve effects on the analysed response variables.

(2.1) Hardness = 0.3371–0.0643A + 0.0387B–0.0300C + 0.0137AB + 0.0103AC + 0.0137BCE – 0.0767A^2^ + 0.0083B^2^ – 0.0605C^2^ + 0.0237ABC +0.3602A^2^B – 0.0158A^2^C

(2.2) Compressive strength = 17.00–0.2500A + 1.0000B–1.50C + 0.0000AB – 3.50AC – 2.00BCE – 2.50A^2^ – 3.50B^2^ – 1.50C^2^

(2.3) Fracture toughness = 0.125000–0.0075A + 0.000025B–0.010000C

(2.4) Brittle Index = 5.74826 + 0A – 0B – 0C

(2.5) Porosity = 49.48 + 0A + 0B + 0C

(2.6) Density = 1.82500 + 0A + 0B + 0C

(2.7) Elastic Modulus = 2.42–0.0388A – 0.3163B–0.3050C + 1.95AB – 1.94AC – 0.8650BCE

### 4.5 Factor and surface response relationship

Fig. 2(a–g) presents a notable alignment between the data and the selected model. The suitability of each model and its adherence to the assumptions of the analyses are assessed through many plots depicting the model's predicted data and the actual data for the trials. Significant disparities were observed between the experimental and projected values for some measured parameters, such as the brittleness index, porosity, and elastic modulus. The observed variations in the brittleness index may be attributed to the experimental determination of hardness values, which are influenced by the indentations made on the pellets. The indentation point has a significant role in determining the level of hardness at a given moment, which might result in the creation of gradients within the datasets. When utilising the acquired datasets for the computation of the brittleness index, it is anticipated that certain deviations may arise. These deviations pertain to the ratio between hardness and fracture toughness. The observed discrepancies in porosity values acquired from experimental data may be attributed to variations in the initial weights of the pellets prior to immersion and subsequent measurements. The sensitivity of nano-indentation measurements for the elastic modulus is considerably high. Furthermore, the indentation point on the pellets holds considerable significance during the process of measurements. These factors may contribute to the discrepancies observed between the actual and projected datasets for the elastic modulus. The heating temperature, denoted as independent variable A, demonstrates a significant influence on the elastic modulus, compressive strength, hardness, and porosity. Similarly, the compaction pressure, represented by independent variable B, demonstrates statistical significance in relation to these important properties.

RETRACTED

**Fig. 2:** Model diagnostic plots of Predicted vs. Actual plot (a) HS, (b) CS (c) FT, (d) BI, (e) PO, (f) DE, and (g) EM.

Fig. 3 displays the interaction plots illustrating the effects of sintering temperature (A) and compaction load (B). Based on the analysis of variance (ANOVA) outcome, it can be shown that Fig. 3 A and B exhibit a significant interaction effect between the sintering temperature and compaction pressure variables in relation to the hardness property. The statistical analysis reveals that the measured hardness value is 0.41 when the sintering temperature is set at 800 °C, the holding period is 1 h, and the compaction load is 500 Pa. The hardness value is affected by the sintering temperature, leading to an increase in the Ca/P ratio [64,65]. Consequently, with the same compaction pressure and temperature, a slightly lower value of 0.36 is obtained, but with an extended duration of 2 h.

**Fig. 3:** Interaction graphs of compaction load and sintering temperature.

Fig. 3C illustrates that the compressive strength value at 500 Pa and 700 °C reached a peak of 12 MPa for both 1 & 2-hr holding times. On the other hand, Fig. 3D provides insight into the probability of obtaining a compressive strength result of 18 MPa. This can be achieved by utilising a sintering temperature of 900 °C with a 1-h holding time and a compaction load of 400 Pa. This graph shows the importance of increasing the sintering temperature due to the preference for higher compressive strength, which is achieved at a lower initial temperature and lower compaction load. Based on the statistical design employed, Fig. 3E and F illustrate the correlation between compaction pressure and sintering in relation to the elastic modulus of the resulting HAp material. The observed trend indicates a significant reduction in elastic modulus with increasing temperature and compaction pressure. At a compaction pressure of 400 Pa and a sintering temperature of 700 °C, the maximum elastic modulus value observed was 4.37 GPa after a holding time of 2 h. Conversely, the lowest elastic modulus value of 0.06 GPa was obtained at a sintering temperature of 800 °C, a compaction pressure of 300 Pa, and a holding time of 2 h. Scaffolds have demonstrated excellent use in tissue engineering due to their elastic modulus values surpassing the critical threshold of 0.06 GPa [35,39]. Fig. 3G and H illustrate the impact of compaction pressure and sintering on the porosity of the resulting hydroxyapatite (HAp) as observed in the statistical design. The observed trend suggests a significant increase in porosity with increasing compaction pressure and holding time, accompanied by a reduction in temperature. With a temperature of 900 °C and a pressure of 300 Pa, the porosity value of 45 % was attained, with the same duration of holding time. Conversely, with a pressure of 500 Pa and a holding period of 1.5 h at 800 °C, a porosity value of 49.5 % was achieved. The observed discrepancies may be attributed to the powder ratio of bovine and catfish bones (39). The observation that the porosity values exceed the established criterion of 49.8 % suggests that these scaffolds possess the potential to be utilised efficiently in the field of biomedical engineering [46,57].

RETRACTED

The study employed response surface (RS) analysis, utilising 2D contour plots and 3D RS plots, to elucidate the interrelationships among the independent factors and their respective effects on the response variables. The data presented in Fig. 4A illustrates the relationship between the compaction pressure (x-axis) and sintering temperature (y-axis) in predicting the hardness of the model. The figure depicts an artificial 3D surface representation of the hardness. At a sintering temperature of 700 °C, it can be demonstrated that the necessary low response values fall within a certain range for compaction pressure. Similarly, at a higher sintering temperature of 900 °C, a lower compaction pressure can be employed to achieve the same outcome. Fig. 4B shows visual responses ascribed to the compressive strength in relation to compaction pressure and sintering temperature, aiming to forecast alterations in compressive strength across different scenarios. However, it is widely accepted in the scientific community that achieving a maximum compressive strength of greater than 11 MPa is possible within a temperature range of 700–900 °C, when subjected to compaction loads ranging from 400 Pa to 500 Pa. Fig. 4C displays the surface representation of the elastic modulus, illustrating the relationship between heating temperature (y-axis) and compaction load (x-axis). The data reveals a decreasing trend in elastic modulus values as the heating temperature decreases from 900 °C to 700 °C. The highest elastic modulus value is observed at a compaction force of 400 Pa. Fig. 4D presents the response values for the surface representation of porosity, with the heating temperature plotted on the y-axis and the compaction load on the x-axis. The observed data shows a decreasing trend in porosity values as the temperature decreases from 900 °C to 700 °C, with the highest porosity value occurring at a compaction load of 300 Pa.

RETRACTED

**Fig. 4:** Hypothetical 3D surface plots of the performance parameters.

The cube plots depicted in Fig. 5 illustrate the interactions between the three elements and the three levels, providing a concise overview of the dynamics in mechanical and physical properties. The increase in holding time and sintering temperature resulted in a decrease in hardness. Similar trends were observed in other characteristics, such as the elastic modulus. The porosity exhibited an increase when subjected to a compaction load of 300 Pa, a holding duration of 2 h, and a temperature of 700 °C. Furthermore, there was an observed increase in the hardness value from 0.37 to 0.45 as the compaction load was increased. The observed trend indicated a positive correlation between the compressive strength and the variables of holding time, sintering temperature, and compaction pressure. The cubic representation of the model exhibiting the minimum projected hardness value of 0.22 GPa is presented in Fig. 5A. This value was achieved by subjecting the model to certain sintering conditions, including a temperature of 900 °C, a compaction load of 400 Pa, and a holding duration of 2 h. Fig. 5B presents cube plots showing the highest projected compressive strength of 17.25 MPa, achieved under the conditions of 900 °C, 500 Pa of CP, and a holding time of 2 h. In Fig. 5C, a cubic representation of the model is depicted, illustrating a high elastic modulus value of 7.235 GPa at a temperature of 800 °C, a holding duration of 2 h, and a compaction pressure of 400 Pa. The cubic representation of the model is depicted in Fig. 5D, illustrating the predicted high porosity data of 43.94 % under the conditions of 700 °C temperature, 2 h holding time, and 300 Pa compaction pressure. These findings are consistent with the references cited as Refs [39,67].

**Fig. 5:** (A)–(D): Cube plots showing the interaction between physical and mechanical properties.

RETRACTED

The best creation of HAp nanoparticles was determined using numerical optimization techniques. This was achieved by evaluating the desirability function, as depicted in Fig. 6, which yielded a value of 0.832. Notably, this value closely approaches unity. The desirability value surpasses the value reported in references [39,46]. Table 6 presents the stated objectives for each response variable, specifically focusing on the reduction of the brittleness index. The lower and upper boundaries for this reduction are set at 4.4 and 7.6, respectively.

**Fig. 6:** Bar charts displaying overall optimized desirability.

**Table 6:** Optimization target for HAp.

Code	Target	Lower boundary	Upper boundary	Lower weight	Upper weight	Prominence
A: Heating temperature	In range	700	900	1	1	3
B: Compaction load	In range	300	500	1	1	3
C: Holding time	In range	1	2	1	1	3
Hardness	Target – 0.305	0.2	0.41	1	1	3
Compressive strength	Target – 13	8	18	1	1	3
Fracture toughness	Maximize	0.04	0.07	1	1	3
Brittle index	Minimize	4.4	7.6	1	1	3
Porosity	Target – 49.51	44.06	54.96	1	1	3
Density	Maximize	1.58	1.89	1	1	3
Elastic modulus	Target – 2.215	0.06	4.37	1	1	3

Table 7 presents the process factors that were optimized to achieve the desired mechanical and physical properties of Hydroxyapatite (HAp). The selected design and mathematical model exhibited a high degree of concordance with the observed values, indicating a strong correspondence between the predicted responses and the actual outcomes. The optimized response exhibits a high degree of agreement with the experimental value of run 6 data, as depicted in Table 3. The bar plot depicted in Fig. 6 illustrates the desirability of each response inside the BBD. The bar graphs illustrate those certain fundamental characteristics, such as porosity, received a comparatively lower ranking in terms of attractiveness when compared to other significant attributes such as hardness, compressive strength, and elastic modulus. However, the practical outcome resulted in an overall optimal solution, which was shown to be highly desirable at approximately 83.2 %. This exceeds the published values in other studies [46,[68], [69], [70]].

**Table 7:** Optimized result.

S/N	Heating temp	Compaction load	Holding time	Hardness	Compressive strength	Fracture toughness	Brittle index	Porosity	Density	Elastic modulus	Desirability
1	837.10	311.73	1.18	0.305	13	0.058	5.74	49.45	1.825	2.216	Selected

Fig. 7a displays the X-ray diffraction (XRD) patterns of the powder prior to the commencement of the experiment, while Fig. 7b exhibits the XRD signatures corresponding to the sample generated during run 6. The main constituent of the given sample was determined to be hydroxyapatite (HAp), which exhibits distinct and strong reflections at a 2θ angle of 21.40, specifically associated with the 211 crystallographic planes. The HAp powders that have undergone complete crystallization exhibit distinct reflections that are clearly observable in both Fig. 7a and b, as referenced in the range of publications from 51 to 55. The characteristic peaks (002, 210, 211, 112, 202, 310, and 222) commonly observed in a standard Hydroxyapatite (HAp) [71,72] are similarly detected in the graphs corresponding to Run 1 (R1) through Run 14 (R14) (Fig. 7 (c) and (d)). This observation suggests that the HAp used in the experiment exhibits a high degree of purity.

RETRACTED

**Fig. 7:** XRD plot of the: (a) HAp powders, (b, c, & d) diagnostic run 6 diagnostic runs 1 - 14.

Additionally, Fig. 8 (a & b) present the Fourier Transform Infrared (FTIR) spectra of the produced Hydroxyapatite (HAp) samples. The obtained samples exhibited prominent peaks in the absorption spectra corresponding to the bonds of PO_4_^3−^ and CO_3_^2−^. These peaks were observed in the wavenumber range of 1000–1500 cm^−1^, and their presence was independent of the powder fraction. The spectra of all samples exhibited minor peaks at approximately 2027 cm^−1^, thereby validating the absence of adsorbed water (O–H) [[15], [73]].

**Fig. 8:** (a &b): FTIR spectra for runs 1-14.

Fig. 9 shows the biodegradability assessment of the diagnostic runs conducted in a phosphate-buffer saline (PBS) solution over a period of 21 days at a temperature of 37 °C. This test was conducted to monitor the degradation of the scaffolds. On the other hand, Fig. 10 illustrates the matching pH values obtained during the experiment. Prior to the gradual decline in weight observed during the incubation period, the scaffold samples exhibited an irregular pattern of weight loss between the time intervals of 2 and 8. A consistent decline was observed from the second day to the fifth day, succeeded by a single-day gain, followed by another consistent decline for one day, and subsequently a slow drop during incubation. It is important to acknowledge the degradability of the generated HAps over time as an indication of their slow solubility or bio-resorbability [74,75]. The data illustrates that the pH levels of the PBS solution exhibited a consistent upward trend across all samples during the initial days. Notably, samples R4, 10, and 14 displayed a considerably greater increase in pH compared to samples R2 and R7, which demonstrated the lowest pH values throughout this time. Subsequently, a persistent decrease in all subsequent runs was observed from day five to day 21. The pH values of runs 4, 6, 12, and 14 showed an initial increase to 10.2 after 5 days, followed by another decrease to 8.6 after 8 days. These pH levels were steady until the 15th day, displaying a consistent trend until the 20th day across all scaffolds. However, on the 21st day, an increase in pH was noted. The high density of HAp can result in the occurrence of microcracks at a pH of 10.2 [76].

RETRACTED

**Fig. 9:** Weight Loss of the diagnostic runs.

**Fig. 10:** (a &b): pH values of the diagnostic runs for 21 days.

The scanning electron microscopy (SEM) pictures of the B100 and C100 samples, as depicted in Fig. 11 (a) and (b) respectively, revealed microstructures characterised by higher density, smaller particle size, and narrower interparticle spacing. These spaces are presumed to be attributable to the presence of pores or voids. The sample composed of a mixture of B50 and C50 (Fig. 11c) as well as the sample obtained from run 6 (Fig. 11d) showed significant presence of large, coarse grains that were frequently densely packed [77]. This observation suggests that the close packing of grains may have influenced the process of densification and the resulting mechanical properties [[48], [49], [50]]. The results obtained from the EDX analysis (which are not displayed) indicate the presence of significant elements, such as calcium, phosphate, magnesium, potassium, strontium, and zinc, in levels that are deemed acceptable, as described in a previous study [78]. The acceleration and enhancement of bone growth and new bone development can be facilitated by the presence of these components in both in vitro and in vivo settings (74).

**Fig. 11:** SEM micrographs of samples B100, C100, B50/C50, and Run 6.

## 5 Conclusion

In this study, HAp nanoparticles were synthesised by a straightforward approach combining direct heat conversion and the sol-gel method. BBED was used as the optimization technique while ANOVA was adopted to evaluate model significance. Out of all variables, the sintering temperature had a remarkable impact on all the target outputs. Furthermore, the density was found to be highly influenced by the duration of holding time, whereas the hardness was observed to be greatly affected by the compaction load. The significance of the interplay between sintering temperature and compaction load was emphasised due to their pronounced influence on the fundamental characteristics of the hydroxyapatite (HAp) scaffolds, namely, hardness, compressive strength, elastic modulus, and porosity. Statistical findings indicate that the sintering temperature, compaction load, and holding period significantly influenced the PO, CS, HS, and EM of the HAp scaffold. The utilisation of restrictions enables the fabrication of HAp scaffolds that exhibit superior mechanical and physical characteristics, hence resulting in anticipated optimized outcomes. The mechanical and physical features of this best-case scenario exhibit a notable similarity to the parameters observed in sample R6. The physical and mechanical properties of the HAp scaffolds were found to be close to their optimal values when subjected to a heat treatment temperature of 900 °C for a duration of 1 h and 18 min, along with a controlled pressure of 311.73 Pa. The X-ray diffraction (XRD) analysis of run 6 revealed that the predominant phase observed in the sample was hydroxyapatite (HAp). The production of the most intense resolved reflections for hydroxyapatite (HAp) commonly occurs at a 2θ value of 21.40, which corresponds to the 211 crystallographic planes. The presence of sharp reflections is a distinguishing feature of a powder that has undergone complete crystallization. Strong peaks were noticed in the absorption bands ranging from 1000 to 1500 cm-1, which relate to the bonds of PO_4_^3−^ and CO_3_^2−^, in the sample labeled as run 6. These peaks were consistently observed regardless of the powder fraction.

RETRACTED

## Data availability statement

Data will be made available on request.

## Additional information

No additional information is available for this paper.

## CRediT authorship contribution statement

**Obinna Anayo Osuchukwu:** Conceptualization, Data curation, Formal analysis, Investigation, Methodology, Visualization, Writing - original draft, Writing - review & editing. **Abdu Salihi:** Formal analysis, Supervision. **Ibrahim Abdullahi:** Formal analysis, Supervision. **Bello Abdulkareem:** Investigation. **Kazeem Adeniyi Salami:** Formal analysis, Software. **Precious Osayamen Etinosa:** Writing - review & editing. **Solomon C. Nwigbo:** Formal analysis, Investigation. **Sikiru Adepoju Mohammed:** Formal analysis, Investigation. **David Olubiyi Obada:** Conceptualization, Data curation, Formal analysis, Methodology, Supervision, Writing - original draft, Writing - review & editing.

## Declaration of competing interest

The authors declare that they have no known competing financial interests or personal relationships that could have appeared to influence the work reported in this paper.
